# Might Patients with Metastatic Gastrointestinal Stromal Tumors Benefit from Operative Management? A Population-Based Retrospective Study

This article has been retracted.

**DOI:** 10.1155/2022/9432410

**Published:** 2022-09-07

**Authors:** Lei Yue, Yingchao Sun, Mengjia Hu, Weiling Hu

**Affiliations:** ^1^Department of Gastroenterology, Sir Run Run Shaw Hospital, Medical School, Zhejiang University, Hangzhou, China; ^2^Department of Gastroenterology, The First Hospital of Jiaxing, Zhejiang, China; ^3^Institute of Gastroenterology, Zhejiang University (IGZJU), Hangzhou, China

## Abstract

**Background:**

With respect to effect of surgery on the therapy of patients with metastatic gastrointestinal stromal tumors (mGISTs), still no consensus has been reached. This research designed to investigate the effect of surgical treatment on prognosis in patients with mGISTs.

**Methods:**

The population-based study consisted of 6282 GIST patients diagnosed between 2001 and 2016, from the Surveillance, Epidemiology, and End Results (SEER) database registry. The Kaplan-Meier method and Cox model were employed for the exploration of the effect of surgery on overall survival (OS) and GIST-specific survival (GSS).

**Results:**

In total, 6282 patients were diagnosed with GISTs, including 1238 (19.7%) mGIST patients and 5044 (80.3%) non-mGIST patients. Compared with the patients with non-mGISTs, metastatic patients assumed relatively lower proportion of surgical management (756 [61.1%] vs. 4666 [92.5%], *P* < 0.001). Based on unadjusted analysis, mGIST patients with operative management presented higher five years OS together with GSS in comparison with those without operative management (OS: 58.3% vs. 33.1%, *P* < 0.001; GSS: 61.6% vs. 36.7%, *P* < 0.001). Multivariable analysis found that no surgery was correlated to more than 2-fold increased death risk (OS, adjusted HR = 2.27, 95% CI: 1.90-2.71; GSS, adjusted HR = 2.42, 95% CI: 2.00-2.93).

**Conclusion:**

Metastatic GIST patients could potentially benefit from operative management with improved GSS and OS.

## 1. Introduction

As the most common mesenchymal neoplasms, gastrointestinal stromal tumors (GISTs) assume a wide range of tumor characteristics ranging from almost inert tumors to rapidly developing tumors. The occurrence of GISTs can involve the whole digestive tract, most commonly in the stomach followed by the small intestine. Almost 4000-6000 new GIST cases were estimated in the US on a yearly basis, and 10-30% of them exhibited clinically malignant [1]. Given that gain-of-function mutation of c-KIT as well as platelet-derived growth factor receptor A (PDGFRA) presented in most GISTs, tyrosine kinase inhibitors (TKIs) have updated and revolutionized the management regimens and prognosis of patients with GISTs [2–4].

At present, the commonly used treatment for localized gastrointestinal stromal tumors is still complete surgical resection. However, 10-15% of GIST patients have overt metastases during initial diagnosis [5, 6]. Metastasis usually occurs in the abdominal cavity or liver, and metastasis to the lung, bone, or brain is rare. Currently, there is no consensus regarding surgical resection of metastatic gastrointestinal stromal tumors (mGISTs) [7–9]. For the lack of effective systemic treatments, resection alone might be the best choice for mGIST patients. Unfortunately, recurrence commonly occurs and majority of patients with liver metastases, for example, relapse within 13 to 17 months [10].

Therefore, Surveillance, Epidemiology, and End Results (SEER) databases were applied for the characterization of the influence of operation on GIST-specific survival (GSS) along with overall survival (OS) in a large population of mGIST patients.

## 2. Methods

### 2.1. Study Population

Data from SEER database was downloaded from 2001 to 2016 for retrospective analysis. As the population-based cancer institution, SEER database covers around 27.8% range of the USA with 18 areas [11]. The SEER data record includes the patients' registration number, personal information, location of the primary lesion, tumor size, tumor code, treatment, and cause of death. International Classification of Diseases for Oncology [ICD-O] cryptogram 8936 was used for the identification of GIST patients.

Figure 1 depicts the flow diagram of patients' selection. Ethical approval and informed consent were exempted by ethics committee on account of the public availability of all the data in SEER database.

### 2.2. Variable Declaration

Demographic features incorporating including race, age at diagnosis, gender, marital status, size, location and grade of tumor, and chemotherapy were extracted from SEER database. Patients were stratified by age of younger (<40 years old) and elder (≥40 years old) [12]. Race was grouped as black, white, some other race (such as Asian/Pacific Islander and American India/AK Native), and unavailable. Marital status was classified as married (consisting of common law), unmarried (including widowed, single, domestic partner, divorced, and separated), and unavailable. ICD-O site was used for identifying tumor sites, which were categorized as the stomach, small intestine, and other digestive organs as well as non-digestive organs. Tumor size was grouped as <2.0 cm, 2.0-4.9 cm, 5.0-9.9 cm, and ≥10 cm. Grade was grouped as poor differentiated or undifferentiated, well or moderately differentiated, or unknown. Chemotherapy was grouped as yes and no/unknown.

### 2.3. Statistical Analysis

Chi-square tests were performed for the comparison of baseline factors for categorical variables between mGIST and non-mGIST patients. Overall vital status and cancer-specific vital status were, respectively, captured in SEER database. Kaplan-Meier analyses were used for detecting between-groups differences of corresponding OS and GSS. In order to eliminate the influence of potential confounding variables, Cox regression analyses were used for developing adjusted HRs (hazard ratios) and pertinent 95% CIs (credibility intervals). Stratification analyses based on different subgroups were conducted for exploring influence of surgery on OS and GSS. *P* value of less than 0.05 was indicative of statistical significance with all *P* being two-sided. SPSS 22.0 was employed for all statistical calculation.

Metastatic GIST patients with exact clinicopathological information were randomly classified into modeling group and validation group (2 : 1). A novel prognostic nomogram was formulated by the rms package in R version 3.6.1 (http://www.r-project.org/) using data from modeling group. Performance of the nomogram was evaluated by Concordance index (C-index) with simultaneous comparison of the predicted value of survival probability by nomogram with Kaplan-Meier observation. Ideally, a good predictive model will have a C-index of >0.70. Calibration curves portrayed the average Kaplan-Meier estimate based on the pertinent nomogram for the 3- and 5-year predicted OS. The bootstrap re-sampling method (1000 repetitions) was used for the acquisition of relatively unbiased estimates and the supervision of interval validation.

## 3. Results

### 3.1. Cohort Characteristics

After a thorough search in the SEER database, we identified 10771 SEER registry patients diagnosed with GISTs from 2001 to 2016. Among these patients, 4489 patients were excluded for the following reasons: bearing multiple primary tumors in 2882, no tissue diagnosis in 107, and insufficient information to analyze in 1500. Finally, a total of 6282 eligible cases including 1238 mGIST patients and 5044 non-mGIST patients were identified. Figure 1 illustrates the flow diagram of patients' selection.

In the mGISTs group, over half (57.9%) were male, while 49.2% were male in the non-mGISTs group. Two groups had a similar mean age (61.1 ± 14.75 vs. 61.1 ± 14.47 years) and an almost equal percentage of adolescents and young adults (≤40 y, 7.4% vs. 7.1%), Caucasian patients (70.4% vs. 67.3%), and married patients (57.0% vs. 57.9%). Compared to the non-mGISTs group, the mGISTs group show less common sites in the stomach (47.3% vs. 61.5%, *P* < 0.001), larger tumor sizes (≥10 cm, 55.8% vs. 25.6%, *P* < 0.001), and a significantly increased proportion of poor differentiated or undifferentiated grade (17.9% vs. 9.3%, *P* < 0.001). Apart from these, mGIST patients were less likely to receive operation (61.1% vs. 92.5%, *P* < 0.001) and more likely to receive chemotherapy (71.4% vs. 35.1%, *P* < 0.001) than non-mGIST patients (Table 1).

### 3.2. Operation in mGIST Patients

Among the 1238 mGIST patients, 756 (61.1%) received surgical management (Table 2). Metastatic GIST patients who had tumors located in the small intestine, with larger size (≥5 cm), or presented as poor differentiated or undifferentiated, were more likely to receive surgery. Female mGIST patients also had more chance of taking surgical management. No major correlations of age, race, or marital status with surgical management of mGISTs were observed.

### 3.3. Prognosis Evaluation

Of mGIST patients, resection group had an apparently higher 5-year GSS (61.6%, 95% CI: 57.7–65.5% vs. 36.7% 95% CI: 31.4–42.0%) than the non-surgery group (Figure 2).

Multivariate Cox regression analysis of the 1238 mGIST patients showed that non-operative management was correlated to a more than 2-fold increased death risk (GSS: HR 2.42, 95% CI 2.00 to 2.93, *P* < 0.001; OS: HR 2.27, 95% CI 1.90-2.71, *P* < 0.001) after the adjustment of age, gender, race, marital status, tumor sites, sizes, grade of differentiation, and chemotherapy. Patients who were older were at higher risk of GIST-specific death (HR: 1.02, 95% CI 1.02-1.03; *P* < 0.001) and overall death (HR: 1.03, 95% CI 1.02-1.04). There was enhanced overall death risk in patients who were unmarried versus those married ones (HR: 1.25, 95% CI 1.06-1.48; *P* = 0.007). Tumor presented and moderately differentiated were at decreased risk of GIST-specific and overall death versus those presented as poor differentiated or undifferentiated (GSS: HR 0.59, 95% CI 0.41-0.85, *P* = 0.004; OS: HR 0.57, 95% CI 0.40-0.80, *P* = 0.001). Besides, we also find that patients with chemotherapy, tumors within the alimentary system, and tumor sizes between and 10 cm were at decreased risk of GIST-specific and overall death (Table 3).

Considering the finding that age at diagnosis, marital status, surgery, chemotherapy, size, location, and grade of tumor were associated with survival outcome, univariate and multivariate COX proportion models were employed between surgery and OS and GSS in subgroup level. Interestingly, in majority of subgroups, we observed that non-surgery was correlated with a more than 2-fold increased hazard of death, which demonstrated that most patients with mGISTs could benefit from surgical managements (Figures 3 and 4). Strikingly, we found that surgery did not improve outcome in patients with tumor size <2 cm (GSS, adjusted HR =2.00, 95% CI: 0.58–7.01; OS, adjusted HR =1.71, 95% CI: 0.54–5.44) (Figure 3 and Table 4).

### 3.4. Novel Prognostic Nomogram for OS Prediction

A total of 336 patients with exact clinicopathological information were randomly classified into modeling cohort (*n* = 224) and validation cohort (*n* = 112) and the characteristics between the two groups were comparable (Table S1). A novel prognostic nomogram that integrated the age, gender, race, marital status, site, size, grade, surgery, and chemotherapy was proposed by multivariate Cox analyses (Figure 5(a)). The C-index for OS-predicting was 0.69 (95% CI: 0.63–0.74) and 0.72 (95% CI: 0.66-0.78) in modeling and validation cohort, respectively. Calibration plot demonstrated that the observed probability of 3- and 5-year OS in the modeling group and validation group presented optimal consistency with the nomogram-predicted OS (Figures 5(b)–5(e)).

## 4. Discussion

Derived from the interstitial cells of Cajal (ICC) and considered the most commonplace mesenchymal carcinomas, gastrointestinal stromal tumors (GISTs) are situated in the digestive tract [13]. The invention of imatinib was a revolution of the treatment of CD117^+^ GIST, which has been the first-line therapy regimen for mGIST patients since 2001 [14]. However, following two years of imatinib therapy, secondary resistance will be presented in approximately half of patients with metastatic or unresectable GISTs [15].

Over the past decade, the function of surgical treatment for metastatic GISTs has expanded. Emerging retrospective studies and rare perspective studies regarding the feasibility of cytoreductive surgery in patients with metastases were performed in American, European, and Asian institutions. For example, several retrospective studies consistently revealed that surgical resection correlated to longer progression-free survival (PFS) and overall survival (OS) in mGIST patients who had preoperative response to TKI therapy [16–19]. Among the few randomized clinical trials evaluating the impact of surgical therapy for mGIST patients, an analysis revealed significantly preferrable OS in the operation cohort compared with the non-operation cohort [20]. Another trial including 41 patients demonstrated that surgical resection of the metastatic lesion potentially improved the prognosis of advanced GIST patients, although there were no significant discrepancies observed between the surgery group (*n* = 19) and imatinib alone group (*n* = 22, 2-year PFS:88.4% vs. 57.7%, *P* = 0.089) [21].

As a population-based database, only SEER is comprehensive in the USA, which consisted of specific survival and treatments information, clinicopathological factors such as disease stage and grade of patients included. Therefore, SEER database is a practically ideal tool to investigating a possible prognosis benefit of surgical management in patients diagnosed as mGISTs in the USA due to the comparative completeness of the data.

In our research, a total of 1238 patients were incorporated from 2001 to 2016 based on SEER database who were diagnosed with mGISTs. These patients were treated in the “real-world” setting compared to those potentially selected patients in most of the clinical trials. Given that the outcome of patients with GISTs dramatically improved after the introduction of tyrosine kinase inhibitors (TKIs) since 2001 [22], we chose to include only mGIST patients diagnosed between 2001 and 2016 in which TKI was prone to widely used for patients with metastatic GIST. We discovered that the use of surgery significantly improved OS and GSS. These results were consistent with those reported retrospective studies [16–19]. As such, patients with metastatic GISTs who meet medical operation indication recommend to conduct resection operation. Potential explanation is the elimination of drug-resistant clones that contribute to not only the possibility of imatinib therapy or other TKIs but also preservation of systemic regimens in the future.

We also found marital status influences the survival of mGIST patients (Table 3). Unmarried patients were at comparably increased risk of presentation with death resulting from mGISTs, regardless the treatment intervention. This phenomenon was observed in the vast majority of cancers [23, 24], which highlights social support potentially has the significant impact on malignant survival. Both tumor sizes and sites—the two best-known risk variables for survival and tumor recurrence—were evaluated in patients with mGISTs in the present study. We observed that patients with tumor between 2 and 10 cm were associated with improved survival versus patients with tumors larger than 10 cm (Table 3). Furthermore, patients with tumor larger than 2 cm could obviously benefit from the operation. However, for those with smaller tumor sizes, the efficacy of surgery was unsupported (Figure 3(a)). Although the number of patients with tumor smaller than 2 cm was small and the conclusion needs to be further validated in large-scale populations, we boldly assume that smaller tumors with distant metastases implies a greater likelihood of malignant behavior and the benefit from surgery may be limited. As for site, we find that the primary foci located in non-digestive system indicate the prognosis is worse than that in the digestive system, which is consistent with previous studies [25].

There were inevitably some limitations in retrospective studies. First of all, the selection bias was introduced due to the lack of detailed information which can equally balance the variables between mGISTs and non-GISTs groups. These variables include specific procedure and site-specific codes for surgery. Therefore, it can hardly draw a conclusion about from whether resecting the primary or metastatic foci that mGIST patients potentially benefit. Future large-scale prospective trials will be vital for clinical decision-making. Furthermore, insufficient information about the regimen, timing, and dosage, responsiveness of chemotherapy, or TKIs, which have significant influence on mGIST progression and survival, also brings a risk of bias. Finally, SEER database lacks information about metastasis foci (distribution, severity), which undoubtedly influences patients' survival. Despite these drawbacks, it is clear to us that surgical management significantly improves GSS and OS in GIST patients diagnosed with metastasis.

In conclusion, operation management correlated to improved OS and GSS in patients with metastatic GISTs. GISTs cannot be thoroughly cured with individual TKIs therapy, and multidisciplinary care is needed to achieve the maximum effect.

## Figures and Tables

**Figure 1:** Flow diagram of the criteria of patients' selection.

**Figure 2:** GIST-specific survival among mGIST patients with surgery management and those without surgery management.

**Figure 3:** GIST-specific survival among mGIST patients with different tumor sizes stratified by surgery management.

**Figure 4:** GIST-specific survival among mGIST patients with different tumor sites stratified by surgery management.

**Figure 5:** (a) mGIST overall survival nomogram. The calibration curve was used for the forecast of patient's survival at (b) 3 years and (c) 5 years in the modeling group and at (d) 3 years and (e) 5 years in the validation group.

**Table 1:** Characteristics of patients with metastatic and non-metastatic GISTs.

Characteristic	Number of patients (%)		*P* value
	Metastatic GIST (*n* = 1238)	Non-metastatic GIST (*n* = 5044)	
Age at diagnosis, y			0.720
<40	91 (7.4)	356 (7.1)	
≥40	1147 (92.6)	4688 (92.9)	
Gender			<0.001
Male	717 (57.9)	2480 (49.2)	
Female	521 (42.1)	2564 (50.8)	
Race			0.036
White	871 (70.4)	3394 (67.3)	
Black	216 (17.4)	891 (17.7)	
Other	146 (11.8)	713 (14.1)	
Unknown	5 (0.4)	46 (0.9)	
Marital status^a^			0.075
Married	706 (57.0)	2919 (57.9)	
Unmarried	487 (39.3)	1874 (37.2)	
Unknown	45 (3.6)	251 (5.0)	
Tumor site			<0.001
Stomach	585 (47.3)	3101 (61.5)	
Small intestine	394 (31.8)	1374 (27.2)	
Other digestive organs	176 (14.2)	377 (7.5)	
Non-digestive organs	83 (6.7)	192 (3.8)	
Tumor size, cm			<0.001
<2.0	41 (3.3)	460 (9.1)	
2.0-4.9	142 (11.5)	1482 (29.4)	
5.0-9.9	364 (29.4)	1810 (35.9)	
≥10	691 (55.8)	1292 (25.6)	
Grade			<0.001
Poor differentiated or undifferentiated	221 (17.9)	470 (9.3)	
Well or moderately differentiated	136 (11.0)	1477 (29.3)	
Unknown	881 (71.2)	3097 (61.4)	
Surgery			<0.001
Yes	756 (61.1)	4666 (92.5)	
No	482 (38.9)	378 (7.5)	
Chemotherapy			<0.001
Yes	884 (71.4)	1768 (35.1)	
No or unknown^b^	354 (28.6)	3276 (64.9)	

^a^Marital status included married (including common law), unmarried (including single, separated, divorced, widowed, or domestic partner), and unknown. ^b^This represents individuals in SEER database with chemotherapy data entered as “No or unknown” was given. It is not possible to separate the true “No” from “true unknown” in the data set. This variable was used because of its importance to survival, despite its limitations.

**Table 2:** Characteristics of metastatic GIST patients stratified by surgical management.

Characteristic	No. (%) of patients		*P* value
	Resection (*n* = 756)	No resection (*n* = 482)	
Age at diagnosis, y			0.503
<40	59 (7.8)	32 (6.6)	
≥40	697 (92.2)	450 (93.4)	
Gender			0.014
Male	417 (55.2)	300 (62.2)	
Female	339 (44.8)	182 (37.8)	
Race			0.073
White	548 (72.5)	323 (67.0)	
Black	115 (15.2)	101 (21.0)	
Other	89 (11.8)	57 (11.8)	
Unknown	4 (0.6)	1 (0.2)	
Marital status			0.495
Married	437 (57.8)	269 (55.8)	
Unmarried	289 (38.2)	198 (41.1)	
Unknown	30 (4.0)	15 (3.1)	
Tumor site			<0.001
Stomach	304 (40.2)	281 (58.3)	
Small intestine	330 (43.7)	64 (13.3)	
Other digestive organs	75 (9.9)	101 (21.0)	
Non-digestive organs	47 (6.2)	36 (7.5)	
Tumor size, cm			<0.001
<2	14 (1.9)	27 (5.6)	
2-4.9	70 (9.3)	72 (14.9)	
5-9.9	227 (30.0)	137 (28.4)	
≥10	445 (58.9)	246 (51.0)	
Grade			<0.001
Poor differentiated or undifferentiated	173 (22.9)	48 (10.0)	
Well or moderately differentiated	120 (15.9)	16 (3.3)	
Unknown	463 (61.2)	418 (86.7)	
Chemotherapy			<0.001
Yes	509 (67.3)	375 (77.8)	
No/unknown	247 (32.7)	107 (22.2)	

**Table 3:** Multivariable analysis of the risk of GSS and OS in metastatic GIST patients^a^.

Variable	GSS		OS	
	Adjusted HR, 95% CI	*P* value	Adjusted HR, 95% CI	*P* value
Surgery				
Yes	1 [reference]	NA	1 [reference]	NA
No	2.42 (2.00-2.93)	<0.001	2.27 (1.90-2.71)	<0.001
Chemotherapy				
Yes	1 [reference]	NA	1 [reference]	NA
No/unknown	1.39 (1.16-1.68)	<0.001	1.47 (1.24-1.74)	<0.001
Age at diagnosis, y	1..02 (1.02-1.03)	<0.001	1.03 (1.02-1.04)	<0.001
Gender				
Male	1 [reference]	NA	1 [reference]	NA
Female	0.90 (0.76-1.07)	0.240	0.87 (0.74-1.02)	0.084
Race				
White	1 [reference]	NA	1 [reference]	NA
Black	0.99 (0.79-1.24)	0.920	1.03 (0.84-1.27)	0.785
Other	0.77 (0.59-1.02)	0.072	0.87 (0.67-1.12)	0.266
Marital status				
Married	1 [reference]	NA	1 [reference]	NA
Unmarried	1.17 (0.98-1.39)	0.086	1.25 (1.06-1.48)	0.007
Tumor site				
Stomach	1 [reference]	NA	1 [reference]	NA
Small intestine	0.93 (0.76-1.15)	0.516	0.92 (0.76-1.12)	0.411
Other digestive organs	1.04 (0.81-1.33)	0.777	1.01 (0.79-1.28)	0.959
Non-digestive organs	1.36 (1.00-1.84)	0.049	1.46 (1.11-1.93)	0.007
Tumor size, cm				
<2	0.81 (0.51-1.28)	0.365	0.86 (0.55-1.32)	0.482
2-4.9	0.66 (0.49-0.87)	0.004	0.69 (0.53-0,.90)	0.006
5-9.9	0.79 (0.65-0.96)	0.016	0.84 (0.80-1.00)	0.054
≥10	1 [reference]	NA	1 [reference]	NA
Grade				
Poor differentiated or undifferentiated	1 [reference]	NA	1 [reference]	NA
Well or moderately differentiated	0.59 (0.41-0.85)	0.004	0.57 (0.40-0.80)	0.001

Abbreviations: NA: not applicable; HR: hazard ratio. ^a^Age at diagnosis and year at diagnosis were included as continuous variables; all other covariates were categorical.

**Table 4:** Association between surgery and OS and GSS among non-metastatic GIST patients in the SEER dataset^a^.

Resection (no vs. yes)	GSS				OS			
	Crude		Adjusted		Crude		Adjusted	
	HR (95% CI)	*P* value	HR (95% CI) ∗	*P* value	HR (95% CI)	*P* value	HR (95% CI) ∗	*P* value
Chemotherapy								
Yes	2.16 (1.76-2.64)	<0.001	2.39 (1.93-2.97)	<0.001	2.17 (1.80-2.64)	<0.001	2.37 (1.93-2.91)	<0.001
No/unknown	2.55 (1.88-3.45)	<0.001	3.13 (2.26-4.32)	<0.001	2.29 (1.73-3.03)	<0.001	2.65 (1.97-3.56)	<0.001
Age at diagnosis, y	2.12 (1.79-250)	<0.001	2.60 (2.17-3.12)	<0.001	2.03 (1.73-2.37)	<0.001	2.44 (2.06-2.89)	<0.001
Marital status								
Married	2.42 (1.93-3.03)	<0.001	2.86 (2.23-3.66)	<0.001	2.36 (1.90-2.93)	<0.001	2.74 (2.16-3.47)	<0.001
Unmarried	1.76 (1.37-2.27)	<0.001	2.23 (1.70-2.94)	<0.001	1.69 (1.34-2.13)	<0.001	2.10 (1.63-2.70)	<0.001
Tumor site								
Stomach	2.36 (1.84-3.02)	<0.001	2.71 (2.08-3.54)	<0.001	2.21 (1.75-2.78)	<0.001	2.53 (1.98-3.24)	<0.001
Small intestine	1.51 (1.01-2.26)	0.043	1.84 (1.18-2.86)	0.007	1.51 (1.03-2.20)	0.033	1.79 (1.18-2.71)	0.006
Other digestive organs	1.69 (1.08-2.62)	0.021	1.96 (1.18-3.25)	0.009	1.62 (1.06-2.46)	0.025	1.78 (1.11-2.87)	0.017
Non-digestive organs	2.12 (1.22-3.69)	0.008	2.37 (1.26-4.45)	0.007	2.15 (1.30-3.55)	0.003	2.39 (1.35-4.26)	0.003
Tumor size, cm								
<2	0.88 (0.36-2.14)	0.782	2.00 (0.58-7.01)	0.275	0.78 (0.34-1.78)	0.558	1.71 (0.54-5.44)	0.363
2-4.9	1.70 (1.00-2.87)	0.048	2.07 (1.19-3.59)	0.010	1.73 (1.07-2.81)	0.027	2.00 (1.20-3.33)	0.008
5-9.9	2.62 (1.90-3.63)	<0.001	3.07 (2.17-4.34)	<0.001	2.42 (1.80-3.26)	<0.001	2.83 (2.05-3.91)	<0.001
≥10	2.37 (1.90-2.96)	<0.001	2.72 (2.14-3.46)	<0.001	2.28 (1.85-2.81)	<0.001	2.57 (2.05-3.22)	<0.001
Grade								
Poor differentiated or undifferentiated	2.66 (1.75-4.05)	<0.001	3.10 (1.99-4.85)	<0.001	2.50 (1.67-3.75)	<0.001	3.00 (1.96-4.61)	<0.001
Well or moderately differentiated	3.35 (1.55-7.22)	0.002	2.68 (1.14-6.32)	0.024	3.38 (1.62-7.03)	0.001	2.72 (1.21-6.15)	0.016

^a^Age at diagnosis and year at diagnosis were included as continuous variables; all other covariates were categorical. ^∗^adjusted for gender, age at diagnosis, race, marital status, site of the tumor, tumor size, chemotherapy and grade of the tumor. OS: overall survival; GSS: GIST-specific survival; GIST: gastrointestinal stromal tumor; SEER: Surveillance, Epidemiology, and End Results.

## Data Availability

All data generated or analyzed during the current study are available from the corresponding author on reasonable request.

## Supplementary Materials

Supplementary Materials Table S1. Characteristics of mGIST patients in training and validation cohorts.
